# Microblog User Emotion Analysis Method Based on Improved Hierarchical Attention Mechanism and BiLSTM

**DOI:** 10.1155/2022/8208561

**Published:** 2022-06-29

**Authors:** Xiao Chen, Xiongliang Xiao

**Affiliations:** School of Electronic Science and Engineering, Hunan University of Information Technology, Changsha, Hunan 410151, China

## Abstract

The goal of Chinese fine-grained emotion analysis is to identify the target words corresponding to fine-grained elements from sentences and determine the corresponding emotional polarity for the target words. Aiming at the problem that the current Sina Microblog user emotion analysis methods have low accuracy and are difficult to effectively predict and manage, a Sina Microblog user emotion analysis method based on the Bidirectional Long Short-Term Memory algorithm (BiLSTM) and improved hierarchical attention mechanism is proposed. Firstly, an emotion analysis model is constructed based on text-level analysis and subjective and objective analysis, and the dimensionality curse problem of one-hot representation is solved by integrating the weighted word vector of TF-IDF. Then, by constructing a bidirectional long short-term memory neural network, the full acquisition of context information is realized, which increases the fine-grained elements of emotion analysis. Finally, by introducing an improved hierarchical attention mechanism, the network model can focus on different parts to achieve text classification and emotion analysis. Through simulation experiments, the proposed emotion analysis method and the other two methods are compared and analyzed under the condition of using the same database. The results show that the precision, recall, and *F*1 value of the method proposed in this paper are the best under 7 different emotion classifications, with the highest reaching 95.8%, 95.9%, and 96.1%, respectively, and the algorithm performance is better than the other two comparisons algorithm. It is proved that the proposed model has excellent performance.

## 1. Introduction

At present, with the deepening of the Internet and social media in people's lives, more and more people use social platforms such as Sina Microblog to convey their various emotions and emotional states [1, 2]. A large amount of text information including the emotions and emotions of different groups accumulated on the network is important data for related user emotion analysis and processing. By analyzing the emotional polarity contained in the text, we can mine valuable information [3]. The text contains a variety of emotional information, and different emotional information expresses the author's different views and attitudes. As a universal social platform, Sina Microblog is loved by more and more people. The emotion expressed by Sina Microblog data is usually not single [4]. For example: “on my birthday, my boyfriend gave me a very beautiful birthday gift. I like it very much. Moreover, my mother made a special school trip to see me. I feel very happy.”. This blog contains two emotions of “like” and “happiness”; that is, the author likes the gifts given by her boyfriend and feels very happy that her mother came to see her. This type of text is usually not a single sentence but consists of multiple sentences [5]. Each or several sentences may express emotional information. Each emotion can be regarded as the emotion tag corresponding to the text, so the text can correspond to multiple tags. Through the reasonable representation and feature extraction of the text, the corresponding multiple tags are regarded as tag information, and the idea of multiple tags is used to solve the problem of emotion analysis.

According to the emotion categories expressed in the mined text, the emotional state of the text publisher can be effectively predicted and managed [6, 7]. In addition, emotional information can also be used as a fine-grained emotional analysis technology to describe the human mental state in a multidimensional way from the perspective of human psychology combined with the traditional coarse-grained emotional analysis [8, 9]. In recent years, text emotion analysis has attracted extensive attention in academia and industry [10].

The remaining sections of this paper are arranged as follows. The second section introduces the relevant research in this field. The third section introduces the user emotion analysis model based on BiLSTM. In fourth section, experiments are designed to verify the performance of the proposed model. The fifth chapter is the conclusion.

## 2. Related Works

The traditional emotion analysis technology is mainly based on single labeling, which cannot analyze a variety of fine-grained emotion information in text data in detail. To solve the recognition of a variety of emotional information contained in the text, it can generally be analyzed as a multilabel classification problem [11–13].

Reference [14] studied the characteristics of public opinion and its evolution over time and proposed an emotional tendency analysis model and obtained the changes of network public opinion characteristics with time series, but this method did not study the prediction process of emotion. Reference [15] describes and calculates the dynamic characteristics of emotion, makes a more comprehensive prediction of the process characteristics describing the evolution of emotion, searches and classifies the information points that allow users to access quickly, and proposes an emotion semantic analysis method based on Wake-Sleep and Support Vector Machine (SVM) method and a deep learning fusion algorithm that can be used for emotion semantic analysis. However, this method cannot be applied to continuous and multidimensional emotional information analysis. Reference [16] proposed a neural network with specific objective emotion analysis because of the long training time of the emotion analysis neural network and the subjective influence of emotion mechanism. However, this method cannot fully obtain context information. Reference [17] takes the relationship between jealousy and EQ as the research object. Through long-term follow-up research on specific populations, longitudinal analysis and cross-lag analysis are carried out on the follow-up results, and the causal relationship between jealousy and EQ is obtained. However, this method has a small scope of application, has certain limitations, and does not give a general emotion analysis method. Reference [18] used the Word2Vec tool to construct an emotion dictionary. On this basis, through a Deep Belief Network and attention model, it constructed and trained the Sina Microblog emotion classification model and proposed a Sina Microblog emotion analysis method based on the dual attention model. However, this method has low accuracy in capturing the relationship between syntactic and semantic words. Reference [19] constructed an emotion dictionary based on seed emotion words and vocabulary similarity calculation method. On this basis, combined with large text data collection and preprocessing and social emotion classification system, it constructed a social emotion analysis model and proposed a hot event emotion analysis method based on an emotion dictionary and text classification method. However, this method only classifies the text emotion into positive and negative attitudes. Reference [20] takes the emotion analysis of Chinese-English mixed texts as the research object, obtains the context semantically related word vector based on the pretraining language model of the large-scale corpus, uses the multilingual attention mechanism to extract the key emotion representations for monolingual and bilingual texts, and proposes a fine-grained emotion analysis model. However, the model convergence speed of this method needs to be improved.

Based on the above analysis, aiming at the problem that the current emotion analysis methods have low accuracy and are difficult to predict and manage effectively, this paper proposes a Sina Microblog user emotion analysis method based on the improved hierarchical attention mechanism and BiLSTM. Compared with traditional emotion analysis methods, the innovation of the proposed method lies in the following:

1. By fusing the weighted word vector of Term Frequency-Inverse Document Frequency (TF-IDF), the cosine distance between vectors can be calculated to represent the semantic distance between words and improve the accuracy of emotion classification.
2. Bidirectional long short-term memory neural network can comprehensively obtain the relevant information of context and analyze the fine-grained emotion.
3. The improved hierarchical attention mechanism can greatly improve the accuracy of emotion classification, thereby improving the overall performance of the model.

## 3. User Emotion Analysis Model Based on AT-BiLSTM

### 3.1. Proposed Model

In this paper, a bidirectional long short-term memory algorithm model based on the improved hierarchical attention mechanism (AT-BiLSTM) is proposed to realize emotion analysis. The algorithm is based on the subjective and objective analysis of sentences and uses the improved hierarchical attention mechanism to focus on the words with strong polarity. The analysis model is established through the network layer of the bidirectional long short-term memory model. The framework flowchart of the proposed AT-BiLSTM algorithm is shown in Figure 1.

Text emotion analysis is divided into word-level analysis, sentence-level analysis, and text-level analysis. The algorithm shown in Figure 1 is based on text-level analysis. In the analysis process, the left-to-right sequence and right-to-left sequence of words in the sentence can be obtained to analyze the similarities and differences of emotion based on the bidirectional double-layer LSTM so that the words about emotion in the words analyzed in the early stage of sentence can effectively affect the analysis results. Secondly, the self-attention mechanism is used to label the obvious special polarity of some words in the sentence, to avoid the probability that sequence analysis may offset the decisive role of some keywords.

### 3.2. Construction of Weighted Word Vector Integrating TF-IDF

The input of the weighted word vector of the fusion TF-IDF consists of the following two parts.

1. The word vector generated by Word2Vec, that is, the word vector represented by one-hot is mapped into the word vector space in an unsupervised way and trained into the form of distributed expression of words. This method solves the problem of dimension disaster in the one-hot representation so that the word vector contains certain semantic information. The words with similar semantics are close in the vector space, and the semantic distance between words can also be expressed by calculating the cosine distance between vectors.
2. TF-IDF weight feature of a word. TF represents word frequency and represents the number of occurrences of a feature word in the corpus. IDF refers to the distribution of a feature word in the corpus. The principle of TF-IDF is that the importance of a feature item in the text database is directly proportional to the number of occurrences of the word in the text database and inversely proportional to the number of texts in the text database. TF-IDF can measure the importance of different features in the text. The Word2Vec word vector feature is fused with the TF-IDF feature based on word frequency statistics to construct the weighted word vector as the input of the model to highlight the words that contribute more to the text emotion classification and improve the accuracy of emotion classification. The specific process is shown in Figure 2.

Firstly, the text to be classified is preprocessed, which mainly includes removing punctuation, removing stop words, and word segmentation of Chinese text. Then, the words obtained by text preprocessing are sorted according to the number of occurrences from high to low, and the words are converted into vector form based on one-hot representation; that is, only the dimension representing the position of the word is 1, and the other dimensions are 0. All words form a dictionary, which is the word direction training corpus. Then the word vector training corpus is sent to the Word2Vec to generate the word vectors based on distributed representation, and the results of text preprocessing are sent to TF-IDF. Assuming that there are *p* comments in the data set and a total of *q* features, and the feature *δ*_*i*_ appears *m* times in the whole data set, the TF and IDF values of this feature are shown in the following formulas, respectively.

(1) $$\begin{array}{c} TF\left(\delta_{i}\right)=\frac{m}{p}, \end{array}$$

(2) $$\begin{array}{c} IDF\left(\delta_{i}\right)=\log\frac{q}{DF\left(\delta_{i}\right)}. \end{array}$$

In formulas (1) and (2), *DF*(*δ*_*i*_) represents the number of comments containing the feature *δ*_*i*_.

The process of calculating the weight *β* of the feature by the TF-IDF method is shown in the following formula.

(3) $$\begin{array}{c} \beta =\frac{m}{p}\cdot \;\log\frac{q}{DF\left(\delta_{i}\right)}. \end{array}$$

On this basis, the weight is normalized, and the weight of each feature word is normalized to be between [0,1]. The process of normalization is shown in the following formula.

(4) $$\begin{array}{c} \beta_{i}=\frac{m/p\cdot \log q/DF\left(\delta_{i}\right)}{\sqrt{m/p\cdot \log q/DF\left(\delta_{i}\right)}}. \end{array}$$

The word vector of *δ*_*i*_ is *a*_*δ*_*i*__, the feature weight *a*_*δ*_*i*__ of *δ*_*i*_ is obtained through the TF-IDF algorithm, and the weight *β*_*i*_ of *δ*_*i*_ is multiplied by the word vector *a*_*δ*_*i*__ of *δ*_*i*_ to construct the weight-based word vector, which is recorded as ${\dot{a}}_{\delta_{i}}$. The process of feature fusion is shown in the following formula.

(5) $$\begin{array}{c} {\dot{a}}_{\delta_{i}}=\beta_{i}\cdot a_{\delta_{i}}. \end{array}$$

### 3.3. BiLSTM

AT-BiLSTM algorithm uses Long Short-Term Memory Model (LSTM) to model text-level text. The overall process is shown in Figure 3.

The artificial neural network with a hierarchical tree structure and the neural network unit recursively processes the input sample characteristics according to the connection order is called Recursive Neural Network, also known as Recurrent Neural Network (RNN). RNN is a kind of multilayer neural network. It takes the sample data set with sequence characteristics as the input sample, evolves, and recurses in the direction of serialization, and all cyclic neural units are connected in a chain. Long short-term memory algorithm (LSTM) is a kind of RNN [21, 22]. LSTM can be used to model temporal data, such as text data. The Bidirectional Long Short-Term Memory model is called BiLSTM for short. The principle of the BiLSTM model is explained from the traditional neural network model.

The goal of fine-grained emotion analysis is to enable the machine to recognize the emotional polarity of different fine-grained elements in a sentence. The goal of Chinese fine-grained emotion analysis is to identify the target words corresponding to fine-grained elements from sentences and determine the corresponding emotional polarity for the target words.

For the fine-grained emotion analysis problem, sometimes the emotion words that affect the fine-grained emotion polarity are in front of the fine-grained element target word, and sometimes the emotion words that affect the fine-grained emotion polarity are behind the fine-grained element target word. For example, “This restaurant has a very clean dining environment, but the food is not delicious.” For the fine-grained element “sanitation,” the emotional polarity word “clean” is in front of the fine-grained element target word “dining environment,” while for the fine-grained element “taste,” the emotional polarity word “not good” is behind the fine-grained element target word “food.” It can be seen that in this kind of problem, the information above should be obtained when judging the emotional polarity. Therefore, this paper constructs the BiLSTM neural network model to fully obtain the context information and then improve the performance of the whole model [23, 24].

The basic structure of BiLSTM is shown in Figure 4.

BiLSTM is composed of two ordinary LSTMs, which can be divided into forward LSTM and reverse LSTM in terms of propagation direction. Unlike ordinary LSTM, BiLSTM does not need to wait until it gets the information of the future. BiLSTM can make the output of the current time node use the information in both forward and reverse directions at the same time. The forward LSTM and the reverse LSTM will not share the state; that is, the output state of the forward LSTM will only be transmitted to the forward LSTM, which has no connection with the reverse LSTM, and the input of the reverse LSTM is the same, and there is no direct connection between them. The input of each time node will be transmitted to the forward LSTM and reverse LSTM, respectively, and then the forward LSTM and reverse LSTM will generate output according to their respective states. Finally, these two outputs are combined as the final output of BiLSTM. The calculation formula is shown in the following formula.

(6) $$\begin{array}{c} o_{t}={\overset{⟶}{o}}_{t}||{\overset{\leftarrow }{o}}_{t}, \end{array}$$

where *o*_*t*_ represents the final output of BiLSTM, ${\overset{⟶}{o}}_{t}$ represents the output result of the forward LSTM, and ${\overset{\leftarrow }{o}}_{t}$ represents the output result of the reverse LSTM.

As can be seen from Figure 4, there is no intersection between the forward LSTM and the reverse LSTM, but they together constitute the output of BiLSTM. Therefore, their contribution to the output of the current time node and the loss caused can be calculated in the training process, and their parameters are also optimized to appropriate values based on the gradient. BiLSTM is very similar to ordinary LSTM in the training process. Two LSTMs have almost no intersection in different directions, so the BiLSTM can be divided into two ordinary LSTMs.

### 3.4. Improve Hierarchical Attention Mechanism

An attribute word may include multiple words. For an attribute word containing *k* words, it can be expressed as *S*={*s*_1_, *s*_2_, *s*_3_,…, *s*_*k*_}, where *s*_*i*_ represents the location index of different words in the attribute word. The hidden layer output corresponding to *S* is represented as *L*={*l*_*s*_1__, *l*_*s*_2__, *l*_*s*_3__,…, *l*_*s*_*k*__} by the corresponding feature vector output by BiLSTM in the previous section. The new vector representation *g*_*s*_ of the attribute word *s* is calculated based on the attention mechanism, as shown in the following formula.

(7) $$\begin{array}{c} g_{s}=\mu L=\sum_{j}\mu_{j}l_{s_{j}}, \end{array}$$

where the sequence of attribute word attention vector *μ*={*μ*_1_, *μ*_2_, *μ*_3_,…, *μ*_*k*_} corresponds to each word of attribute word *S* in turn. The attention vector *μ* is the self-attention vector calculated by using the hidden layer output as the input; that is, the input feature vector comes from the output result of the upper layer language model. The calculation of *μ* is shown in the following formula.

(8) $$\begin{array}{c} \mu =\text{softmax}\left[\omega_{a2}\tanh\left(\omega_{a1}L\right)\right], \end{array}$$

where *ω*_*a*1_ ∈ *R*^*d*_*k*_×*d*_*l*_^ and *ω*_*a*2_ ∈ *R*^1×*d*_*l*_^ are parameters of the attention mechanism.

After paying attention to the key points of the internal words of attribute words, it is necessary to refine the attention of each specific attribute word in all words of the whole sentence. The vector representation sequence used is still the hidden output of the upper layer, but the global sentence-level attention will use the feature vector *C* of each word in the sentence with length *L*_0_={*l*_1_, *l*_2_, *l*_3_,…, *l*_*C*_}. Sentence-level attention is also based on the linear combination of hidden layer output to obtain a single vector, as shown in the following equation.

(9) $$\begin{array}{c} g_{m,s,a}=\lambda L=\sum_{i}\mu_{i}l_{i}, \end{array}$$

where *λ*={*λ*_1_, *λ*_2_, *λ*_3_,…, *λ*_*C*_} represents the sentence-level attention vector and *λ*_*i*_ encodes the attention of each word in the sequence about attribute word *S* and aspect *a*.

In the process of calculating *λ*, firstly, *l*_*i*_ is transformed into a vector representation of *d*_*k*_ dimension by using the multilayer neural network of tanh activation function and then put into SoftMax to generate the probability distribution of the sequence, as shown in the following formula.

(10) $$\begin{array}{c} \lambda =\text{softmax}\left[g_{a}^{S}\tanh\left(\omega_{k}\left(L⊙g_{s}\right)\right)\right]. \end{array}$$

where *g*_*s*_ represents the word vector of aspect and *L*⊙*g*_*s*_ represents the concatenation of *g*_*s*_ and each *l*_*i*_. *ω*_*k*1_ ∈ *R*^*d*_*k*_×*d*_*l*_^*d*_*k*_ is to map the row vector of *L* to the *d*_*k*_-dimensional space, and *ω*_*k*2_ ∈ *R*^1×*d*_*l*_^ maps each new row vector to an unnormalized attention weight.

The objective function of the training classifier is to minimize the sum of the accumulated cross-entropy loss of the predicted attribute word aspect, as shown in the following formula.

(11) $$\begin{array}{c} G=\frac{1}{\left|D\right|}\sum_{T\in D}\sum_{s\in T}\sum_{a\in A}\log\;p_{b,s}^{a}, \end{array}$$

where *A* represents the predefined aspect set, *p*_*b*,*s*_^*a*^ is the probability that the emotional polarity is predicted to be *b* under the conditions of aspect *a* and attribute word *s*. It is calculated using the SoftMax function, as shown in the following formula.

(12) $$\begin{array}{c} p_{b,s}^{a}=\text{softmax}\left(\omega^{\left(1\right)}g_{m,s}+\rho_{m}^{a}\right). \end{array}$$

Here, *ω*^(1)^ and *ρ*_*m*_^*a*^ represent the parameters of the affective polarity prediction tag for the aspect *a* to which attribute word *s* belongs.

### 3.5. Loss Function

The training of the proposed model adopts the end-to-end backpropagation mode, and the loss function adopts the cross-entropy loss function. The formula is shown in the following formula.

(13) $$\begin{array}{c} \text{LOSS}=-\sum_{\left(m,a\right)\in D}\sum_{c\in C}p_{m,a}^{g}\left(c\right)\log\left[p_{m,a}\left(c\right)\right], \end{array}$$

where *D* represents the training data set. *C* represents the category of emotion classification. The value of 1 or 0 for *p*_*m*,*a*_^*g*^(*c*) indicates whether the polarity of the correct emotion is predicted. *p*_*m*,*a*_(*c*) represents the probability (*m*, *a*) predicted by the model that belongs to the category *C*. The gradient of all parameters is calculated using the backpropagation algorithm. All parameters are randomly initialized, and they satisfy the normal distribution *U*(−0.01,  0.01). The stochastic gradient descent (SGD) algorithm is used to update the parameters, and the supervised learning method is used for the training of the whole model.

## 4. Experiments and Analysis

### 4.1. Experimental Data Acquisition and Operation Environment

The experimental data is obtained for the mobile terminal of Sina Microblog. The data acquisition is mainly based on the Scrapy crawler framework, which collects the Sina Microblog comment data of 7 cases that have attracted much attention in recent years from the Sina Microblog platform, requests the Sina Microblog API to return JSON format data, and parses it through the JSON module in Python to obtain the desired data. The main fields and meanings of Sina Microblog comments are shown in Table 1.

Through the above process, the corresponding Sina Microblog user comment data is finally obtained. Among them, there are 11264 *A* events, 12597 *B* events, 18341 *C* events, 15675 *D* events, 30247 *E* events, 39648 *F* events, and 57634 *G* events, a total of 185406 events. After the completion of data acquisition, according to the different needs of emotion classification tasks and emotional reasons for data, the Sina Microblog comment emotion classification data set and Sina Microblog comment emotional reasons data set are constructed, respectively.

To construct the Sina Microblog user comment emotion classification data set, it is necessary to manually label the Sina Microblog comment data. The emotion label adopts seven emotions defined in the emotional vocabulary of Dalian University of Technology, which are happiness, like, anger, sadness, fear, evil, and surprise. Comments that do not contain emotions will not be considered, and comments that contain emotions will be marked as one of the above seven emotions. Specifically, 35000 comments were randomly sampled from the obtained Sina Microblog comment data for manual annotation. The annotation work was completed by three people, and only the data with consistent annotation was retained. To keep the annotation data of each emotion category balanced, 2000 annotation data of each category are selected. Finally, the Sina Microblog comment emotion classification data set is obtained. The statistical information of the data set is shown in Table 2.

The operating environment of the experiment is shown in Table 3.

### 4.2. Evaluating Indicator

The experiment uses the precision (*P*), recall (*R*), and *F*1 value (*F*1) in NLPCC2013 Chinese Sina Microblog emotion analysis and evaluation as the evaluation indicator. Their calculation methods are shown in the following formulas, respectively.

(14) $$\begin{array}{c} P=\frac{S_{T}}{S}, \end{array}$$

(15) $$\begin{array}{c} R=\frac{S_{T}}{S_{G}}, \end{array}$$

(16) $$\begin{array}{c} F1=2\cdot \frac{P\cdot R}{P+R}, \end{array}$$

where *S* represents the number of submitted results, *S*_*T*_ represents the number of matches with manual annotation in the submitted results, and *S*_*G*_ represents the number of manual annotation results.

### 4.3. Analysis of Experimental Results

In the training set and validation set, the loss value and accuracy of the AT-BiLSTM algorithm proposed in this paper are calculated, and the results are shown in Figure 5.

As can be seen from Figure 5, the loss of the training set is decreasing with the increase of the number of training iterations, while the loss of the validation set does not decrease significantly, which shows that the model performs well in the training set but does not have generally high prediction accuracy in the validation set. Since this experiment mainly analyzes the comment data set of Sina Microblog users, the model parameters of the last iteration of the validation set can represent the performance of the test set Sina Microblog user comment data set.

### 4.4. Comparative Analysis

The following is a comparative analysis of the method proposed in this paper and the methods in [14, 15]. The precision, recall, and *F*1 value of different analysis methods under the same data set are calculated, and the results are shown in Figures 6–8, respectively.

It can be seen from Figures 6to 8 that when the same data set is used, the emotion analysis method proposed in this paper is better than the other two comparison methods in three evaluation indicators. The precision, recall, and *F*1 value are the highest in seven different emotions, reaching 95.8%, 95.9%, and 96.1%, respectively, and the lowest are 93.6%, 93.7%, and 94.1%, respectively. The results show that the weighted word vector fused with TF-IDF can effectively solve the problem of dimensionality disaster and improve the accuracy of emotion classification. BiLSTM can comprehensively obtain context information to improve the recall of emotion analysis. The improved hierarchical attention mechanism can improve the precision of emotion classification. This is because the introduction of the weighted word vector of the fusion TF-IDF makes the word vector contain certain semantic information. Words with similar semantics are relatively close in the vector space. By calculating the semantic distance between words and highlighting words that contribute more to text emotion classification, the precision and recall of emotion classification are improved.

## 5. Conclusion

In view of the low accuracy of current Sina Microblog user emotion analysis methods and the difficulty of effective prediction and management, this paper proposes a Sina Microblog user emotion analysis method based on BiLSTM and an improved hierarchical attention mechanism. The dimension disaster problem is solved by using the weighted word vector fused with TF-IDF. Construct a bidirectional long short-term memory neural network to fully obtain the context information. An improved hierarchical attention mechanism is introduced to achieve accurate classification. Future work will focus on further research to explore the cross-representation methods of different emotional causes and emotion analysis methods when different emotional causes interact.

## Figures and Tables

**Figure 1:** Framework flowchart of AT-BiLSTM algorithm.

**Figure 2:** Construction process of weight-based word vector.

**Figure 3:** Process for modeling text-level text using long short-term memory network.

**Figure 4:** The basic structure of BiLSTM.

**Figure 5:** Loss and precision of AT-BiLSTM algorithm.

**Figure 6:** Precision of different algorithms under 7 emotions.

**Figure 7:** Recall of different algorithms under 7 emotions.

**Figure 8:** *F*1 values of different algorithms under 7 emotions.

**Table 1:** Main fields and meanings of Sina Microblog comments.

Field	Meaning
Case	The event this comment belongs to
User	User who commented
Comment	User's comments
Date	The date of user comment

**Table 2:** Statistics of the data set.

Emotional label	Data set
Happiness	2000
Like	2000
Anger	2000
Sadness	2000
Fear	2000
Disgust	2000
Surprise	2000
Sum	14000

**Table 3:** Experimental operating environment.

Name	Model
Operating system	Linux Ubuntu-X299-UD4-Pro 4.15.0-47-generic x86_64 GNU/Linux
CPU	Intel® Core™ i7-7800X 3.50 GHz ∗12
GPU	GeForce GTX 1018 Ti *∗*2
Python	Python 3.6.7
Keras	Keras 2.2.4
TensorFlow	TensorFlow 1.13.1

## Data Availability

The data used to support the findings of this study are included within the article.
